# Informatization of Accounting Systems in Small- and Medium-Sized Enterprises Based on Artificial Intelligence-Enabled Cloud Computing

**DOI:** 10.1155/2022/6089195

**Published:** 2022-08-12

**Authors:** Jingjie Zhao, Liming Zhang, Yue Zhao

**Affiliations:** ^1^School of Management, Jilin University, Changchun 130022, China; ^2^Changchun Polytechnic, Changchun, Changchun 130028, China

## Abstract

Against the backdrop of China's growing market economy, small- and medium-sized enterprises (SMEs) have taken advantage of this opportunity to develop rapidly. At present, SMEs have become an important part of the market economy. Accounting system information management system is an advanced form of management, and improving the degree of accounting information is the key to improving the management mode of SMEs. This study applies cloud computing to enterprise accounting management systems. The results show that realizing SME accounting information management can effectively improve economic settlements. With the development of cloud computing, its improvement of accounting management efficiency cannot be ignored. Besides, the risks of accounting informatization, enterprises can make their development by establishing a secure network protection wall and relying on strict relevant laws and regulations.

## 1. Introduction

Nowadays, with the help of the rapid development of big data technology, enterprises are getting better and better and can handle a lot of tedious things. However, there are still some areas that need to be improved, especially the hidden dangers of information security and the risk of information management. Therefore, it is necessary to improve the enterprise accounting information work. Only in this way can the development of the accounting industry be more stable, and at the same time, the emerging technology of big data can be developed more maturely, and the development of each enterprise can be more long term [1]. However, in the face of rising costs, small- and medium-sized enterprises hope to use information technology to solve problems, build enterprise information systems at low cost, and achieve integration with external information systems. Cloud computing uses a flexible business billing method, which makes it a highly attractive and platform support for the application of information technology to small- and medium-sized enterprises. If the small- and medium-sized enterprises can use the cloud computing platform to establish their own enterprise accounting information system, accounting information will play a greater role in the business activities of enterprises [2]. The main function of this model is that related computing resources can be configured in the network, and visitors can freely mobilize related services, such as network, server, storage device, application program and other related services, according to their own requirements. These resources are quickly sent to the hands of demanders and announced in a timely manner, which reduces the usual management costs to a minimum and reduces the interference and interference caused by service providers. Cloud computing has contributed its own strength to accounting informatization, and is an inevitable path in line with the development of modern informatization [3].

The emergence of artificial intelligence brings new opportunities and challenges to accounting informatization. The application of artificial intelligence technology in accounting work will greatly improve the efficiency of accounting work and the accuracy of accounting information, and provide a strong boost for the development of enterprise accounting informatization. The rapid development of the Internet has spawned new products such as cloud computing. Subsequently, the development of cloud computing has promoted the development speed of the Internet. At the same time, cloud computing has gradually developed into an important means for small- and medium-sized enterprises to maintain their own development. Small- and medium-sized enterprises can reasonably use the characteristics of cloud computing to build an accounting informatization model. Relying on the environment of cloud computing, small- and medium-sized enterprises have a clear direction and advanced means for the reform of accounting information. Through a comprehensive and systematic understanding of cloud computing, and a correct and objective study of cloud computing, small- and medium-sized enterprises are conducive to building a scientific, practical, and efficient accounting informatization model [4].

With the development of the times, the amount of information has increased sharply, and the original information technology can no longer process and analyze the massive data, and cloud computing is born. The concept of cloud computing was proposed by foreign companies such as *IBM* and Amazon, and then cloud computing was added to the application of information systems. Companies such as Google and Microsoft provide platform services for the application of cloud computing in the field of accounting informatization. Chyzhevska et al. [5] used various cutting-edge technologies such as embedded systems, mobile networks, mobile computing, cloud computing, big data, data analysis technology, and embedded cloud computing to analyze accounting and finance. It proves that it is a feasible solution to apply cloud computing to accounting informatization. In terms of cloud computing service technology, European and American countries have always been at the leading level, and the application of cloud computing is also quite extensive. In terms of security protection of cloud computing services, the technologies and regulations of European and American countries are quite mature, and they are in a leading position in the world, representing the development level of cloud computing service security, and it is worth learning from many countries [6–9]. As shown in Figure 1, there are many factors that affect the accounting system, of which technology and policies have a huge impact. From the initial simple informatization construction to the current accounting informatization that has the function of supporting decision-making, the accounting informatization construction in China has only experienced several decades. After the emergence of cloud computing, many enterprises began to introduce cloud computing in accounting informatization, and built a cloud computing accounting service platform to promote the intelligence of accounting informatization. However, at present, the development of accounting informatization based on cloud computing is not mature, and it is still in the development stage, but the inevitable trend of accounting informatization construction in the future.

The development of informatization of enterprise accounting system using cloud computing in China is the adaptation and development of the times, and informatization management is an important way of modern enterprise management. Compared with other methods, cloud computing has a greater advantage in the construction of accounting informatization for small- and medium-sized enterprises. As shown in Figure 2, this paper also points out the current constraints of small- and medium-sized enterprises in the construction of cloud computing informatization, including the use of various funds mentioned in the figure. Based on this, an effective implementation model of the national level, the operator level and the enterprise level are proposed to solve the problem of path selection for the development of accounting informatization in small- and medium-sized enterprises under the cloud computing technology environment [10–12]. The greatest highlight of this study is the application of cloud computing to the accounting and settlement system of SMEs, which realizes the information management of SMEs' accounting and effectively improves the efficiency of economic settlement. The improvement of accounting management efficiency in this study is not negligible.

## 2. Feasibility Analysis of Accounting System Informatization under Cloud Computing and Artificial Intelligence

At the beginning of the last century, the huge domestic market gap and potential demand drove the rapid development of large enterprises. The traditional computerized financial information processing model has been unable to meet the needs of the actual operation of enterprises. It is mainly manifested in the fact that traditional computing is oriented to the financial department, and the process from financial information processing to decision-making is still too cumbersome and the cycle is too long compared to reality [13, 14]. Artificial intelligence can use image recognition, voice recognition, and other technical means to convert written financial information into virtual data and save it in electronic equipment, which avoids a lot of time and energy when manually preparing financial statements and reports, makes daily clearing business more convenient, and can make corresponding accounting treatment according to specific accounting objects and working characteristics, it has higher timeliness and pertinence [15]. Today, e-commerce platforms are gradually taking the center stage, and the value of data is infinitely amplified, which is called the era of big data. In short, “big data” refers to a multicategory dataset composed of a large amount of data, the data content of which cannot be collected and processed by traditional database tools. From this, the “cloud computing” model and the arrival of the entire cloud era are derived [16]. These resources can be deployed quickly and require little administrative effort or interaction with service providers. Cloud computing is essentially a service, not a technology. As shown in Figure 3, the growth of information system utilization efficiency over time shows a trend of peaks. The so-called service is to focus on the actual needs of users, rather than from the perspective of technical implementation or management personnel to look at cloud computing. According to the needs of users, cloud computing platform service providers provide customers with corresponding service platforms or service programs, and customers use the corresponding cloud computing services to complete their own information system construction work [17].

The accounting model using cloud computing mainly involves basic information facilities such as data resources and network storage. It also requires servers such as servers that provide computer capabilities, management platforms, and application software that participate in the development of various accounting services. Therefore, it is necessary to make full use of the existing conditions and create an information-based accounting system that belongs to the small- and medium-sized enterprises [18].

The development of accounting information system has the development characteristics of all systems. With the continuous integration of information systems, the data generated are also increasing. When playing the role of the information system, it is necessary to introduce cloud computing technology to better utilize the system through virtualization and high reliability of cloud computing. At present, the information system based on cloud computing is an inevitable trend of development. As a part of the system, the accounting information system will follow the development trend of the system and introduce cloud computing technology to build an accounting information system based on cloud computing. Therefore, the development of accounting informatization based on cloud computing is an important manifestation of the application of system theory [19].

Small- and medium-sized enterprises in China have disadvantages such as financing difficulties, lack of high-level talents, and limited decision-making ability of enterprises. The foundation and process of accounting informatization are not as valued and invested by large enterprises. As shown in Figure 4, the simulation curve of the algorithm shows a gradually rising state. With the in-depth development of market economy construction, the efficiency of computer accounting has become more apparent. The emergence of cloud computing technology, due to its low participation threshold and low price, is a small- and medium-sized enterprise. The development of accounting informatization provides the possibility [20].

The big data cloud computing model is a revolutionary change for small- and medium-sized enterprises, which brings new ideas. In the financial system, a leap-forward development has been achieved. First, enterprises do not need to invest in equipment construction, which is extremely important for small- and medium-sized enterprises whose available funds are often insufficient. Secondly, the construction of informatization has improved the efficiency of enterprise management by enterprise decision makers. Artificial intelligence can also use the ability of storage and location analysis to deeply study financial data, and build a database within the enterprise to solve various difficult problems. In addition, artificial intelligence technology can also process the financial and accounting data in real time, so that the leadership can control the financial dynamics in real time. Artificial intelligence technology can also reengineer business processes according to accounting information, and can also improve accounting efficiency. The systems for financial management in the modern market economy environment. Small- and medium-sized enterprises can choose a cloud model that suits them according to their own characteristics and business scope.

## 3. Effective Way of Application of Cloud Accounting Information System for Small- and Medium-Sized Enterprises

### 3.1. Use *SaaS* Service Platform to Improve Management Capabilities

The use of SaaS platform to carry out accounting informatization construction of small- and medium-sized enterprises is a very effective way for small- and medium-sized enterprises to improve their management capabilities. The biggest advantage of the *SaaS* application model is the use of service leasing. The enterprise connects the user's *PC* to the *SaaS* operating platform through the Internet, and the enterprise adopts the *SaaS* service model for accounting informatization construction. Through the *SaaS* platform, customers can enjoy a complete set of informatization conveniences such as server, network, system administrator, online office management, financial management, etc. As shown in Figure 5, online and offline distribution is more scattered, which not only saves the cost of accounting information application but also enables users to obtain the convenience and convenience brought by advanced technology. Fast, and at the same time, it can improve the management ability of the enterprise itself. Using the SaaS platform, small- and medium-sized enterprises can use the least capital and spend the least energy to build the most suitable accounting information management system for the enterprise itself [21, 22].

(1) $$\begin{array}{c} EC\left(cpu\right)=A\times B\times C\times \left(C-c\right)\times VM. \end{array}$$

In the ideal case, the power consumption of the memory is a linear function of time.

Under the cloud computing model, small- and medium-sized enterprises can obtain professional consulting and the latest technology applications provided by large service providers, so that the efficiency of business process reorganization and accounting management of small- and medium-sized enterprises can be improved. In addition, due to the openness and sharing of the Internet, cloud service providers are supervised by many users, which will make them devote more energy to creating higher satisfaction and service levels in a fiercely competitive environment [23, 24].

### 3.2. Increase the Application of Virtualization Technology According to the Actual Situation

Virtualization can reduce the *IT* cost of enterprises and save more human resource costs from personnel. Because personnel only need to maintain a few physical equipment instead of maintaining each *PC*. In terms of hardware, enterprises can virtualize a large number of virtual devices that can be actually used by using few hardware devices. In terms of software, administrators only need to install software on the virtual machine once, and then they can virtualize to all devices, and at the same time, it will bring great convenience when software upgrades [25–27].

(2) $$\begin{array}{c} n_{ij}=x_{i}^{\min}+r\left(x_{j}^{\max}-x_{i}^{\max}\right), \end{array}$$

where *x*^max^ and *x*^min^ represent the minimum and maximum values of the *j*-th dimension elements of all available food sources in the global search space, respectively. *r* is a random parameter between 0 and 1.

Another benefit of virtualization is higher service assurance levels at a lower cost. *IT* maintenance operations such as backup and recovery can be performed quickly using virtualization technology. As shown in Figure 6, the cluster configuration or high reliability deployment, and the use of virtualization can simplify and improve the reliability of server deployment, patch management, configuration updates, backup, security, auditing and compatibility, and reduce service management time.

When small- and medium-sized enterprises start to create an accounting information system, they need to standardize the accounting information system in advance. First of all, *SMEs* should have a clear understanding and careful control of their own situation. The establishment of accounting information system needs to understand the accounting management requirements of the enterprise, the development goals of the enterprise, the economic capacity of the enterprise, and the development scale of the enterprise. These factors will have a great impact on the accounting information of the enterprise. For promoting the construction of the accounting information system, it is necessary to master and consider these details. Secondly, through the collection, arrangement, and analysis of various data, scientific and detailed specification of the construction of the accounting work information system are carried out.

(3) $$\begin{array}{c} \phi =\sum_{i=1}^{j}\sum_{m}\alpha_{i}^{j}, \end{array}$$

where *α* represents the deployment decision of virtual machine *i* to mobile device *j*, and *i* is a natural number.

### 3.3. The Problem of Data Conversion and Integration between Heterogeneous Platforms

With the continuous growth of the scale, the *SaaS* platform used at this time can no longer need enterprises. At the same time, as shown in Figure 7 the data of small- and medium-sized enterprises are also growing, its risk also increases, do not want to put their key private data on a third-party service platform. At this time, the enterprises will choose to build their own separate accounting information system within the enterprise, but they will face a problem: how to migrate the data previously run on the *SaaS* platform to the system they built? Some basic data can be downloaded and imported into the new system through the export function of the *SaaS* platform. However, some very personalized business data often cannot be exported from the *SaaS* platform, and such problems often lead to incoherent business data for small- and medium-sized enterprises [28]. Figure 7 shows the comparison between network security risks and other security risks

(4) $$\begin{array}{c} w_{i}=\frac{n_{i}\mathrm{\times Α}{Ν}_{i}}{\sum_{j=1}^{m}n_{i}\mathrm{\times Α}{Ν}_{j}}, \end{array}$$

where the weight of mobile devices in all devices and the mobile device community is *w*_*i*_.

When they initially choose cloud computing platforms for accounting informatization construction, they should focus on the problems of data migration and integration in the future. As shown in Figure 8, the capital reserve situation has become smaller over time, and the personnel reserve is also regionally stable. In addition, the corresponding service providers can be required to issue the platform data interface specifications and standards to clarify whether the data can be smoothly migrated from the cloud platform if the *SMEs* build their own accounting information systems. Based on cloud computing technology, the engineering settlement cloud computing platform optimizes the engineering settlement audit process and improves audit efficiency and audit accuracy. As Figure 8 shows, it is very beneficial to establish an efficient project settlement cloud platform based on cloud computing.

In addition, cloud computing has also improved the application efficiency. Because the accounting information system of the cloud computing model is constructed through the Internet, enterprise users can obtain the required services only through the Internet in the process of use. The collection and inquiry of informatized accounting information enables the accountants of the enterprises to inquire and inspect the account information anytime and anywhere, and can also grasp the latest business data released by the enterprise anytime and anywhere. At the same time, the platform interaction function provided by cloud computing can help mutual aid enterprises to carry out faster decision-making and enterprise management control. For small- and medium-sized enterprises with cross-regional or multinational business, accountants located in different regions can operate online at the same time and carry out collaborative work, which improves the efficiency of the enterprises' accounting informatization work.

## 4. Risk Analysis of Artificial Intelligence and Cloud Computing in Accounting Informatization

Company *A* is a new type of medium-sized management financial enterprise. Its main businesses include fund management, automatic identification technology products such as radio frequency identification, and mobile terminal products. The company was established in Hangzhou in 2015. After years of development, the company has grown to 380 employees. Three subsidiaries were set up in Hefei, Nanchang, and Wuhan, and the company's business has been affirmed in the fields of infrastructure and hotels.

(5) $$\begin{array}{c} R_{i}^{j}=\frac{\sum_{\delta \in sma}TM_{m}}{w_{i}}. \end{array}$$

In this formula, under the premise of the solution vector *s*, the value of *R*_*i*_^*j*^ is proportional to the division processing time.

Company *A* does not have an accounting information summary system, and all information statistics are done by manpower. Then the accuracy of the accounting information submitted cannot be guaranteed, so that the accounting analysis cannot easily detect the problem. As a result, it cannot effectively improve the management level of company *A*.

(6) $$\begin{array}{c} T_{\min}=\min_{s\in S}T_{s}, \end{array}$$

where *T* represents the minimum total processing time of all |*S*| candidate solution vectors.

Issues such as those listed above lead to additional costs for companies to rearrange information during the final aggregation step. At the same time, the process of sorting out the data takes a period of time, which is more obvious when the scale is larger. Therefore, from the perspective of the results, it takes a long process to finally aggregate the data, which forms a time delay, and the value of the information itself is further reduced. Furthermore, the processing of data not only takes time but the time spent by the company is also included in the cost of the company. Moreover, there may be some errors in the reprocessing of data, which greatly affects the timeliness of decision-making.

(7) $$\begin{array}{c} E\left(X\right)=\sum_{i=1}^{N}X_{i}\times p\left(x_{i}\right). \end{array}$$

This formula represents the calculation formula of cloud computing mathematical expectation.

In the whole system of the company, Company *A* needs to play the role of financial monitoring. However, due to the geographical distance of the subsidiaries, it is impossible for Company *A* to monitor the generation and processing of every information of the subsidiaries in real time. In the form of spot checks. After random inspection, a series of accounting problems often occur in subsidiaries, such as credits in asset accounts, debits in liability accounts, errors in the provision of depreciation in the current month, errors in the calculation of exchange gains and losses at the end of the month, incorrect value of inventory at the end of the period or errors in cost carry-forward.

(8) $$\begin{array}{c} d\left(x_{\alpha },x_{\beta }\right)=\sqrt{\sum_{i=1}^{m}\left(x_{\alpha i},x_{\beta i}\right)}. \end{array}$$

This formula is the Euclidean distance to measure the similarity of two data objects *x*_*αi*_ and *x*_*βj*_.

In the artificial intelligence environment, accounting information is collected, processed, and saved in digital form. Compared with traditional information means, virtual information is easier to be destroyed and stolen. Enterprises should pay timely attention to the development of artificial intelligence industry, prepare development plans according to their own capabilities, select influential professional companies in the industry for system development and maintenance, and effectively ensure the accuracy and timeliness of accounting information management. In response to the above problems of company *A*, the cloud computing method is used to correct them. Because the biggest feature of the *SaaS* model information system is that the operation can be completed directly on the browser without installing a series of software. Therefore, a certain workload is reduced in the product trial process. During the trial, it was found that its online access speed is fast, its service is relatively stable, its operation is simple and convenient, and its after-sales service quality is good [29]. Due to the rapid development of the company's business, and showing the characteristics of variability, it may be necessary to change the function of the system from time to time in the process of informatization. Therefore, the company must maintain communication with the cloud service provider at any time. When there is a business demand that needs to change the module function, it will jointly complete the improvement and upgrading of the system with the cloud service provider. Through preliminary attempts, company A mainly adopts the two core modules of “online accounting” and “online purchase, sales and inventory” in the network system to build the company's information system platform, which will introduce more service operations according to the actual needs.

## 5. Analysis on Risk Factors of Enterprise Accounting Informatization

Enterprise accounting information system from the perspective of big data plays a more and more important role in enterprise development.  Figure 9 is a schematic diagram of the basic components of cloud computing. It can improve the accounting business level of enterprises, reduce the burden of accounts, and improve the accounting analysis data, but at the same time, with the increase of application modules, it increases the cost of accounting information system maintenance and the risks in the use process. Therefore, the attention of enterprise management must be improved.

A high degree of security is the most important aspect of an accounting system. To sum up, there are three main problems in the current enterprise accounting information system under the big data platform: First, the stability of the operating system of the big data sharing platform is weak. Second, the system has loopholes in identity security management. Third, the database encryption method is flawed. These potential risk factors will bring huge economic losses to enterprises and hinder the further development of accounting information systems.  Figure 10 shows the structure of the accounting information system for SMEs. These problems are mainly caused by the construction of the big data resource sharing platform of the accounting information system, the security of the platform, and the imperfect matching laws and regulations [30].

(9) $$\begin{array}{c} Z_{t}=\sum_{i=1}^{N}w_{m}e^{-ayC\left(x\right)}. \end{array}$$

The algorithm in the above formula can continuously reduce the training error during the training process, that is the classification error rate on the training dataset.

(10) $$\begin{array}{c} Q_{s}=e^{-\left(1/m\right)\sum_{j=1}^{m}\sum_{q=1}^{r_{j}}\left(PS_{q}-PD_{q}\right)\log\left(PS_{q}/PD_{q}\right)}, \end{array}$$

where *PS*_*q*_ represents the proportion of samples in *S* that take the *q*-th feature attribute value on feature *j* from the sampling dataset *S*.

Security is the most critical part of an accounting information system. It is used to maintain the normal operation of all aspects of the accounting system. Once there is a problem with the security of the system, it will threaten the normal operation of the enterprise. According to the survey, nearly 60% of enterprises refuse to use the network platform to store and calculate enterprise accounting information and management data. Mainly due to concerns about identity security authentication and database encryption technology loopholes, this not only means that the security of the network system is poor but it also means that the construction of China's information security platform is not sound.

(11) $$\begin{array}{c} f\left(x\right)=\sum_{i=1}^{M}T\left(x;\theta_{i}\right), \end{array}$$

Where *θ*_*i*_ represents the model parameters and *T* represents the decision tree model.

## 6. Accounting Informatization Path Selection and Countermeasure Analysis

In the cloud computing technology environment, how to promote the accounting informatization of small- and medium-sized enterprises is a complex task involving many aspects including the country, the operation service, and the enterprise itself. Only by following the inherent laws of its own development, actively participating in various aspects, and forming work synergy, can it achieve its healthy and orderly development.

(12) $$\begin{array}{c} r_{g}^{k}=\eta \times \max\left[d\left(x_{i},G_{k}\right)\right]. \end{array}$$

Among them, *η* can take values such as 0.2, 0.3.

In the process of cloud computing service application and promotion, it is an important basic task to eliminate the hidden security risks of information and data to the greatest extent, and it is also the biggest restrictive factor affecting the enthusiasm of small- and medium-sized enterprises to adopt cloud computing services. In the cloud computing accounting information system, there are unified regulations for accounting documents, accounting methods, subject settings, and internal codes. This unified model can reduce accounting conflicts between different departments. In order to make the enterprise accounting informatization security system more perfect, building a network firewall can improve the security of the system and better protect the accounting informatization data from being leaked. The financial operation management services provided by the big data cloud computing platform have gradually improved the development requirements of small- and medium-sized enterprises. For the consideration of input-output ratio and the pursuit of corporate profits, most small- and medium-sized enterprises are more inclined to obtain high-end services such as financial analysis, forecasting, and information decision-making for the purpose of purchasing cloud computing services. Cloud computing service operators should face the constantly escalating service demands of customers, continuously strengthen technological innovation, develop cloud computing service modules, expand and extend service fields, and improve service quality and level. This study can be served as a continued work to former research of the application mode of financial informatization in enterprises based on data mining. In this study, the settlement process varies greatly between accountants in different years and regions, and the results are not satisfactory. Through the construction of accounting cloud computing platform, a unified engineering settlement process can be established to increase the standardization and work efficiency of business and thus improve the settlement level of enterprises.

## 7. Conclusion

Cloud computing is a new domain, although its development process is relatively short, its impact is huge and far reaching. Its incomparable technical advantages and significant cost advantages provide a favorable development opportunity for small- and medium-sized enterprises to solve their informatization problems in terms of capital, technology, talents, etc. Enterprises in the era of big data can have better development space, but there are also many adverse effects. Especially when using big data and cloud computing, there will be some security risks and information management risks. These risks are now handled with better preventive measures. In particular, for the risks of accounting informatization, enterprises can make their own development in the era of big data smoother and safer by establishing a secure network protection wall and relying on strict relevant laws and regulations.

This paper discusses in detail how to promote the popularization and application of cloud computing services in the current accounting informatization construction of small- and medium-sized enterprises. Mainly through the current status of the development of accounting informatization in small- and medium-sized enterprises, the accounting informatization in the cloud computing environment is introduced, and its application value is analyzed. Then, by comparing with the traditional accounting informatization, and the real application case of company A, try to put forward a framework scheme for small- and medium-sized enterprises to apply cloud computing services for accounting informatization construction. And how to promote the popularization of cloud computing services in the application of accounting informatization in small- and medium-sized enterprises, from the perspectives of the country, the operator, and the enterprise itself, it puts forward specific and feasible countermeasures and suggestions. The complexity of cloud-based computing results in a significant decrease in the performance of scheduling algorithms. The future work direction can be based on this problem for in-depth research.

## Figures and Tables

**Figure 1:** Contribution of various factors to the system.

**Figure 2:** The use of various fees in the cloud computing model.

**Figure 3:** Information system utilization efficiency.

**Figure 4:** SaaS calculates simulated values.

**Figure 5:** Online accounting and invoicing value chart.

**Figure 6:** Percentage of operating modes in each year.

**Figure 7:** The size of the impact of different hazards.

**Figure 8:** Schematic diagram of reserve conditions at different stages.

**Figure 9:** The basic components of cloud computing.

**Figure 10:** Structure diagram of accounting information system for small- and medium-sized enterprises.

## Data Availability

The data used to support the findings of this study are available from the corresponding author upon request.
